The article "Targeting the Vav3 oncogene enhances docetaxel-induced apoptosis through the inhibition of androgen receptor phosphorylation in LNCaP prostate cancer cells under chronic hypoxia" was published in 2013. Journal: Mol Cancer.

# Targeting the Vav3 oncogene enhances docetaxel-induced apoptosis through the inhibition of androgen receptor phosphorylation in LNCaP prostate cancer cells under chronic hypoxia

**DOI:** 10.1186/1476-4598-12-27

**Published:** 2013-04-08

**Authors:** Takeo Nomura, Mutsushi Yamasaki, Kenichi Hirai, Toru Inoue, Ryuta Sato, Keiko Matsuura, Masatsugu Moriyama, Fuminori Sato, Hiromitsu Mimata

**Affiliations:** 1 Department of Urology, Oita University Faculty of Medicine, 1-1 Idaigaoka, Hasama-machi, Yufu, Oita 879-5593, Japan; 2 Department of Molecular Pathology, Oita University Faculty of Medicine, 1-1 Idaigaoka, Hasama-machi, Yufu, Oita 879-5593, Japan

**Keywords:** Vav3, Docetaxel, Androgen receptor, Prostate cancer, Chronic hypoxia

## Abstract

**Background:**

The Vav family of Rho/Rac guanosine nucleotide exchange factors comprises three members in mammalian cells. Vav3 enhances androgen receptor (AR) activity during progression to androgen independence in prostate cancer. We examined Vav3 small interfering RNA (siRNA) effects on cell proliferation and apoptosis in docetaxel-treated LNCaP cells under chronic hypoxia (LNCaPH).

**Methods:**

We examined individual and combined effects of Vav3 siRNA (si-Vav3) and docetaxel on cell growth and apoptosis under chronic hypoxia by cell proliferation, flow cytometric, DNA fragmentation, and immunoblot analyses. To clarify the molecular basis of si-Vav3- and docetaxel-induced apoptosis, we analyzed alterations in phosphatidylinositol 3-kinase (PI3K)/Akt, extracellular signal-regulate kinase (ERK), c-jun N-terminal kinase (JNK), and AR pathways using kinase inhibitors in LNCaPH cells. The effects of si-Vav3/atelocollagen complex alone or in combination with docetaxel were assessed on xenografts in nude mice by tumor growth delay.

**Results:**

Vav3 overexpression was observed in LNCaPH compared with the expression under normoxia. Interrupting Vav3 signaling using siRNA enhanced docetaxel-induced cell growth suppression compared with that induced by docetaxel alone by inhibition of Akt and ERK phosphorylation, resulting in AR phosphorylation inhibition. In addition to increased B-cell lymphoma 2 (Bcl-2) phosphorylation through JNK signaling in response to docetaxel, si-Vav3 enhanced docetaxel-induced apoptosis, as characterized by the accumulation of sub-G1 phase cells and DNA fragmentation, through Bcl-xL/Bcl-2-associated death promoter (Bad) dephosphorylation, resulting in increased caspase-9, caspase-3, and cleaved poly(ADP-ribose) polymerase activation. Xenograft tumor growth was slightly inhibited by si-Vav3/atelocollagen complex injection and combined use of si-Vav3/atelocollagen complex and docetaxel produced a greater effect than docetaxel alone.

The article "Targeting the Vav3 oncogene enhances docetaxel-induced apoptosis through the inhibition of androgen receptor phosphorylation in LNCaP prostate cancer cells under chronic hypoxia" was published in 2013. Journal: Mol Cancer.

**Conclusions:**

Interrupting Vav3 signaling enhances docetaxel-induced apoptosis in LNCaP cells under chronic hypoxia by inhibiting the PI3K/Akt, ERK, and AR signaling pathways. Therapy targeting Vav3 in combination with docetaxel may have practical implications for managing castration-resistant prostate cancer.

## Background

Prostate cancer is the most frequently diagnosed cancer in the world. Most prostate cancers are initially dependent on androgens for growth, and patients with prostate cancer receive hormonal therapy. Androgen deprivation by medical or surgical castration contributes significantly to disease control during early stages of prostate cancer; however, the effect is usually palliative, and a majority of prostate cancers eventually progress to a hormone-refractory phenotype against which current treatments are relatively ineffective [1]. The progression of prostate cancer from the androgen-dependent to androgen-independent state is the main obstacle in improving the survival and quality of life in patients with advanced prostate cancer. Therefore, much attention has been focused on the evolution from androgen-dependent to androgen-independent prostate cancer, and the establishment of novel therapeutic strategies against hormone-refractory prostate cancer (HRPC) is desirable.

In the past, molecular mechanisms for the progression to the hormone-refractory state have been proposed based on experimental evidence. The androgen receptor (AR)-dependent mechanisms include (a) androgen-independent activation of AR [2,3], (b) AR overexpression or mutations, which could allow AR to respond to lower levels of androgens [4] or be directly activated by other ligands [5], (c) increased expression of steroidogenic enzymes [6], and (d) indirect activation of AR by cell-surface receptors such as HER2 [7], the interleukin-6 receptor [8] and G-protein-coupled receptors [9]. The AR-independent mechanisms include (e) mutations of tumor suppressor genes [10], (f) expression of various oncogenes affecting cell growth and death [11], (g) enhanced angiogenesis [12], (h) bypassing the AR pathway [13], and (i) prostate cancer stem cell regeneration [14].

Recently, Lyons *et al*. reported a novel ligand-independent AR activation through Rho guanosine triphosphatase (GTPase) signaling in prostate cancer *in vivo* and *in vitro *[15]. The levels of Vav3, a Rho GTPase guanine nucleotide exchange factor (GEF), are elevated in human prostate cancer specimens, and they increase during the progression of prostate cancer to androgen independence by enhancement of AR transcriptional activity [16,17]. The Vav gene (Vav1) was first identified in hematopoietic cells with oncogenic activity. Since the discovery of the Vav oncogene, new family members have been identified in mammalian cells (Vav2 and Vav3) [18-20]. The biochemical functions of Vav family proteins have been extensively investigated. Vav1 expression is restricted to hematopoietic cells, and it is involved in the formation of the immune synapse. Vav2 and Vav3 are more ubiquitously expressed [20]. Vav proteins contain the Dbl homology domain, which confers GEF activity, as well as protein interaction domains that allow them to function in pathways regulating actin cytoskeleton organization [21]. In particular, their GEF activity is the most important function among them. Vav3, a signal transducer of receptor protein tyrosine kinase, is involved in various cellular signaling processes including cell morphology modulation and cell transformation with oncogenic activity [22]. In the current study, Vav3 was demonstrated to bind to phosphatidylinositol 3-kinase (PI3K), leading to PI3K activation with cell transformation activity [23].

The article "Targeting the Vav3 oncogene enhances docetaxel-induced apoptosis through the inhibition of androgen receptor phosphorylation in LNCaP prostate cancer cells under chronic hypoxia" was published in 2013. Journal: Mol Cancer.

In a previous report, *Dong et al.* found that Vav3 enhances AR activity partially through PI3K/Akt signaling and stimulates androgen-independent growth in prostate cancer [17]. We further revealed that tumor cell hypoxia induced Vav3 overexpression with androgen-independent growth and malignant behavior in LNCaP cells [24,25]. Therefore, we hypothesized that Vav3 has an important role in regulating the growth and survival of prostate cancer cells under hypoxic conditions and that it is a novel therapeutic target for the treatment of HRPC. In recent years, taxane-based chemotherapy has contributed to improvements in treatment outcomes in prostate cancer, and docetaxel has become a standard chemotherapeutic agent for treating HRPC; however, docetaxel does not exhibit sufficient activity when administered as a single agent [26-28]. However, when docetaxel is used in combination with other therapeutic modalities, this therapeutic strategy may provide meaningful improvements in the management of HRPC. In this study, we report studies assessing *in vitro* and *in vivo* combinations of docetaxel with small interfering RNA (siRNA) for Vav3.

To the best of our knowledge, we have reported for the first time that interrupting the Vav3 signaling pathway using siRNA induces apoptosis and enhances docetaxel sensitivity through the inhibition of PI3K/Akt, extracellular signal-regulate kinase (ERK), and AR signaling axis in human prostate cancer.

## Results

### Expression levels of Vav3 in parental and chronic hypoxic LNCaP cells

The expression of Vav3 was assessed by immunoblot analysis and immunocytochemistry in parental LNCaP cells (LNCaP) and LNCaP cells cultured under hypoxic conditions for over six months (LNCaPH). Compared with LNCaP cells, LNCaPH cells and KPK13 cells as positive control expressed higher levels of Vav3 (Figure 1A and B).

The article "Targeting the Vav3 oncogene enhances docetaxel-induced apoptosis through the inhibition of androgen receptor phosphorylation in LNCaP prostate cancer cells under chronic hypoxia" was published in 2013. Journal: Mol Cancer.

**Figure 1:** **Expression of Vav3 in LNCaP, LNCaPH, and KPK13 cells. A**, immunoblot analysis of cell lysates derived from LNCaP, LNCaPH, and KPK13 cells. M. W., Molecular weight. **B**, immunocytochemical staining of Vav3 in LNCaP, LNCaPH, and KPK13 cells.

### Effects of si-Vav3 and docetaxel on Vav3 expression and cell proliferation in LNCaPH cells

Because Vav3 increased LNCaP cell growth *in vitro* and Vav3 overexpression was observed in LNCaPH cells exhibiting androgen-independent behavior compared with its expression in LNCaP cells [24,25], we tested the possibility that Vav3-induced intracellular signaling may be a therapeutic target for the treatment of HRPC. LNCaPH cells were transiently transfected with either si-Vav3 or si-Scr. After 72 h, cells were harvested and subjected to immunoblot analysis, revealing that si-Vav3 effectively downregulated the expression of Vav3 compared with its control expression (Figure 2A). Conversely, Vav3 expression was unaffected by docetaxel treatment.

**Figure 2:** **Effects of Vav3 siRNA (si-Vav3) and docetaxel (DTX) on cell proliferation and Akt, ERK, and JNK activation in LNCaPH cells. A**, Vav3 siRNA (si-Vav3) and control scramble siRNA (si-Scr) were added to the medium using a lipophilic transfection-enhancing reagent (Lipofectamine RNAiMAX) in the presence or absence of DTX. Cells were harvested after 72 h, and immunoblot analysis was performed using anti-Vav3 antibody. Blots were stripped and reprobed with an antibody against β-tubulin. **B**, effects of si-Vav3 in the presence or absence of DTX on the proliferation of LNCaPH cells were determined by cell counting. Values represent the mean ± SE of three independent experiments. Asterisk indicates P <0.05 compared with LNCaPH cells treated with DTX alone. **C**, live/death viability/cytotoxicity kit assay was used to detect live (green) and dead (red) cells using fluorescence microscopy (4× magnification). **D**, phosphorylation of Akt, ERK, and JNK induced by si-Vav3 in the presence or absence of DTX was determined by immunoblot analysis using phospho-Akt (Ser 473), phospho-ERK (Thr 202/Tyr 204), and phospho-JNK (Thr 183/Tyr185) antibodies. Blots were stripped and reprobed with antibodies against total Akt, total ERK, total JNK, and β-tubulin. **E**, phosphorylation levels of Akt, ERK, and JNK in LNCaPH cells were scored as 1.00, and each value is shown as a fold stimulation. Values represent the mean of three independent experiments. Asterisk indicates P < 0.05 compared with LNCaPH.

The article "Targeting the Vav3 oncogene enhances docetaxel-induced apoptosis through the inhibition of androgen receptor phosphorylation in LNCaP prostate cancer cells under chronic hypoxia" was published in 2013. Journal: Mol Cancer.

To determine the docetaxel sensitivity of si-Vav3-treated cells, cells transfected with si-Vav3 or si-Scr were treated with 5 nM docetaxel for 72 h and assayed for cell proliferation and live/death analyses. Treatment with docetaxel or si-Vav3 inhibited cell growth in a time-dependent manner, and when LNCaPH cells were treated with si-Vav3 in the presence of docetaxel, sensitivity to docetaxel was significantly enhanced (P < 0.05) (Figure 2B). We further confirmed this enhanced cell growth inhibition with the results of the cell live/death assay. The assay stains live cells with a green fluorescence dye and dead cells with a red fluorescence dye. We observed that control si-Scr and si-Vav3 treatment resulted in the death of 0.5% and 8% of cells respectively, whereas treatment with docetaxel alone or si-Vav3 plus docetaxel resulted in the death of 48% and 78% of cells per field, respectively (Figure 2C). These results suggest that Vav3 depletion significantly sensitizes LNCaPH cells to docetaxel treatment by inducing cell death.

### Effects of si-Vav3 and docetaxel on the activation of Akt, ERK, and JNK signaling in LNCaPH cells

To clarify the molecular mechanisms by which si-Vav3 and docetaxel promote the death of LNCaPH cells, we investigated the effects of si-Vav3 and docetaxel on the phosphorylation of Akt, ERK, and JNK. LNCaPH cells were treated with si-Vav3, 5 nM docetaxel, or si-Vav3 plus 5 nM docetaxel for 48 h. Treatment with si-Vav3 led to the attenuation of Akt phosphorylation at Ser 473, a site required for Akt activation, and ERK phosphorylation at Thr 202 and Tyr 204, which are sites required for ERK activation, but no effect was observed on JNK phosphorylation (Figure 2D). Similarly, docetaxel treatment attenuated Akt and ERK phosphorylation and strongly induced JNK phosphorylation at Thr 183 and Tyr 185, which are sites required for JNK activation (Figure 2D). When LNCaPH cells were treated with si-Vav3 plus docetaxel, Akt phosphorylation was completely abolished with the inhibition of ERK phosphorylation and JNK activation (Figure 2D). Figure 2E summarizes the results of three independent experiments. These results suggest that LNCaPH cells display Akt and ERK activation and that si-Vav3 negatively regulates PI3K/Akt and ERK pathway activation, enhancing the effects of docetaxel.

### Effects of si-Vav3 and docetaxel on the apoptotic cell death of LNCaPH cells

To investigate whether the growth-inhibitory effects of the combination of si-Vav3 and docetaxel may be triggered by increased apoptosis in LNCaPH cells, we evaluated the apoptotic cells by flow cytometry, which assessed a sub-G1 population of apoptotic cells, and enzyme-linked immunosorbent assay (ELISA) using Cell Death Detection ELISA^PLUS^. Treatment with 5 nM docetaxel led to increased apoptosis in LNCaPH cells in a time-dependent manner, but the sub-G1 population was slightly increased by si-Vav3 alone. When LNCaPH cells were treated with si-Vav3 plus docetaxel, a strong induction of apoptosis was observed (Figure 3A). Similarly, the addition of si-Vav3 to docetaxel markedly induced apoptosis in a docetaxel concentration-dependent manner (Figure 3B). Among cells treated with si-Vav3 plus 5 nM docetaxel for 72 h, 42.4, 9.0, 10.8, and 37.8% of cells were in the sub-G1, G1, S, and G2/M fractions, respectively (Figure 3C). In LNCaPH cells treated with si-Vav3 or 5 nM docetaxel for 24 h, 7.3 and 19.6-fold increases in DNA fragmentation, respectively, were recorded, but combination treatment resulted in a 40.2-fold increase in DNA fragmentation compared with the untreated control (Figure 3D). These results are consistent with the significant growth inhibition of LNCaPH cells induced by si-Vav3 plus docetaxel, and these combined effects were associated with a large increase in the number of apoptotic cells.

The article "Targeting the Vav3 oncogene enhances docetaxel-induced apoptosis through the inhibition of androgen receptor phosphorylation in LNCaP prostate cancer cells under chronic hypoxia" was published in 2013. Journal: Mol Cancer.

**Figure 3:** **Effects of Vav3 siRNA (si-Vav3) and docetaxel (DTX) on apoptosis and Bcl-2, Bad, and AR activation in LNCaPH cells. A**, **B**, **C** and **D**, si-Vav3 in the presence or absence of DTX induced apoptosis in LNCaPH cells, as detected and quantified by flow cytometry and DNA fragmentation. Note the percent of apoptotic cells with sub-G1 DNA content and fold increase in DNA fragmentation. LNCaPH cells were treated with or without si-Vav3 in the presence or absence of 5 nM DTX for the indicated times (**A**) or DTX at the concentrations of 0, 1, 2.5, and 5 nM for 72 h (**B**). Values represent the mean ± SE of three independent experiments. Asterisk indicates P <0.05 compared with LNCaPH cells treated with DTX alone. **C**, change in the cell cycle distribution in response to si-Vav3 in the presence or absence of DTX for 72 h. **D**, detection of apoptotic cells using Cell Death Detection ELISA^PLUS^ following 24-h treatment with si-Vav3 in the presence or absence of 5 nM DTX. Values represent the mean ± SE of three independent experiments. Asterisk indicates P < 0.05 compared with LNCaPH cells treated with DTX alone. **E**, caspase-9 and caspase-3 activation and PARP cleavage after treatment with si-Vav3 in the presence or absence of DTX for 72 h. Blots were stripped and reprobed with an antibody against β-tubulin. LNCaP cells were treated with 10 nM DTX (a known apoptosis inducer) for 72 h as a positive control for apoptosis. *F*, Bcl-2, Bad, and AR phosphorylation induced by si-Vav3 in the presence or absence of DTX was determined by immunoblot analysis using phospho-Bcl-2 (Ser 70), phospho-Bad (Ser 112), and phospho-AR (Ser 81) antibodies. Blots were stripped and reprobed with antibodies against total Bcl-2, total Bad, total AR, and β-tubulin.

The article "Targeting the Vav3 oncogene enhances docetaxel-induced apoptosis through the inhibition of androgen receptor phosphorylation in LNCaP prostate cancer cells under chronic hypoxia" was published in 2013. Journal: Mol Cancer.

Because apoptosis can be triggered by death receptor-mediated or mitochondria-mediated cascades depending on the type of caspase activation, we evaluated caspase-8, caspase-9, and caspase-3 activation and subsequent cleavage of PARP engaged in DNA repair in LNCaPH cells treated with si-Vav3, 5 nM docetaxel, or si-Vav3 plus 5 nM docetaxel for 48 h. Immunoblot analysis revealed that si-Vav3 or docetaxel alone induced the activation of caspase-9 and caspase-3 and cleavage of PARP, respectively. When LNCaPH cells were treated with si-Vav3 plus docetaxel, we observed enhanced caspase-9 and caspase-3 processing and PARP cleavage (Figure 3E). In this series of experiments, we did not observe any activation of caspase-8 (data not shown). To clarify the extent of caspase and PARP cleavage in LNCaPH cells, these results were compared with those in LNCaP cells treated with 10 nM DTX (a known apoptosis inducer) for 72 h. These results collectively provide supportive evidence that treatment with si-Vav3 enhances docetaxel-induced apoptosis primarily through a mitochondrial pathway.

To further elucidate the molecular mechanisms underlying si-Vav3- and docetaxel-induced apoptosis of LNCaPH cells, we investigated the Bcl-2 family proteins and AR, which are known to be regulated by PI3K/Akt, ERK, or JNK signaling. We observed that the levels of Bcl-2 phosphorylated at Ser 70, but not the total levels of Bcl-2 protein, were increased by docetaxel compared with in the level of control (nontreated or si-Scr-transfected) cells, whereas the levels of Bad phosphorylated at Ser 136 but not total levels of Bad protein were decreased by treatment with si-Vav3 and docetaxel. In addition to Bcl-2 family activation, si-Vav3 decreased the levels of AR phosphorylation at Ser 81, but molecular events were not affected by docetaxel (Figure 3F). These results suggest that si-Vav3- and docetaxel-induced apoptosis is regulated by the activation of Bcl-2, Bad, and AR through independent pathways in LNCaPH cells.

### AR phosphorylation depends on the activation of PI3K/Akt and ERK signaling in LNCaPH cells

To determine whether inhibition of selected survival pathways is sufficient to induce apoptosis, we used pathway-specific inhibitors of Akt, ERK, and JNK signaling in parental LNCaP and LNCaPH cells. The effects of LY294002 (PI3K inhibitor), U0126 (mitogen-activated protein kinase inhibitor), and SP600125 (JNK inhibitor) on apoptosis were examined by flow cytometry. In these experiments, serum-starved cells were treated with LY294002 (25 μM) or U0126 (20 μM) alone or together for 48 h. LY294002 or U0126 alone increased the percentage of apoptotic cells compared with the control (DMSO-treated) cells in both LNCaP and LNCaPH cells (Figure 4A). The combined use of LY294002 and U0126 promoted cell death, but their effects were not additive because the levels of ERK phosphorylation were not high compared with those of Akt phosphorylation in both LNCaP and LNCaPH cells (Figure 4A and B). LNCaP cells were less sensitive to LY294002 compared with LNCaPH cells because the phosphorylation level of Akt was lower in LNCaP cells than in LNCaPH cells, but the effects of U0126 in LNCaP and LNCaPH cells were equivalent because the phosphorylation level of ERK was similar in both cell lines. In contrast, when cells were treated with SP600125, we observed no change in the percentage of apoptotic cells in both LNCaP and LNCaPH cells (Figure 4A).

The article "Targeting the Vav3 oncogene enhances docetaxel-induced apoptosis through the inhibition of androgen receptor phosphorylation in LNCaP prostate cancer cells under chronic hypoxia" was published in 2013. Journal: Mol Cancer.

**Figure 4:** **Effects of specific kinase inhibitors on select signaling pathways and apoptosis in LNCaP and LNCaPH cells.** LNCaP and LNCaPH cells were pretreated with 25 μM LY294002, 20 μM U0126, and 10 μM SP600125 alone or the combination of LY294002 and U0126 for 48 h. Control cells were grown in the presence of DMSO. **A**, note the percent of apoptotic cells with sub-G1 DNA content. Values represent the mean ± SE of three independent experiments. Asterisk indicates P < 0.05 compared with LNCaP cells. **B**, immunoblot analysis was performed using antibodies that specifically recognize total and phosphorylated Akt, ERK, JNK, and AR. Blots were stripped and reprobed with an antibody against β-tubulin.

To further evaluate whether PI3K/Akt, ERK, and JNK signaling pathways affect AR phosphorylation, we performed immunoblot analysis using pathway-specific inhibitors. The AR phosphorylation level was higher in LNCaPH cells than in LNCaP cells. LY294002 or U0126 alone weakly decreased AR phosphorylation at Ser 81 in LNCaPH cells, but when these two inhibitors were added simultaneously, we found that AR phosphorylation was completely abolished (Figure 4B). In contrast, AR phosphorylation was strongly inhibited by LY294002 or U0126 alone due to the lower phosphorylation level of AR in LNCaP cells. The level of phosphorylated AR was associated with the induction of apoptosis in both LNCaP and LNCaPH cells (Figure 4A and B). These results suggest that Vav3 enhances the phosphorylation of AR at Ser 81 through PI3K/Akt and ERK pathways in LNCaPH cells. When LNCaP and LNCaPH cells were treated with SP600125, no alteration in AR phosphorylation was observed (Figure 4B). This result indicates that JNK is an independent signaling component and its signaling does not converge with PI3K/Akt and ERK, which affect the phosphorylation of AR in both LNCaP and LNCaPH cells.

The article "Targeting the Vav3 oncogene enhances docetaxel-induced apoptosis through the inhibition of androgen receptor phosphorylation in LNCaP prostate cancer cells under chronic hypoxia" was published in 2013. Journal: Mol Cancer.

### In vivo antitumor activity of si-Vav3 alone and in combination with docetaxel

We first assessed the dose–response relationship of si-Vav3/atelocollagen complex therapy to optimize the effects of si-Vav3. The effects of si-Vav3 depended on the amount of the si-Vav3/atelocollagen complex, but the difference in the effects of si-Vav3 between 2.5 μg and 10 μg of the siRNA/atelocollagen complex was not large (Figure 5A). Therefore, we selected 2.5 μg of si-Vav3/50 μl/tumor as the optimal concentration for combination therapy with docetaxel. In our preliminary studies, the docetaxel dose of 20 mg/kg maximally suppressed tumor growth without significant toxicity in mice. Therefore, we chose 10 mg/kg as a suboptimal dose in the subsequent studies. The tumor growth curves shown in Figure 5B demonstrate that the growth-inhibitory effect of si-Vav3 alone was weak, but the combination of si-Vav3 and docetaxel was highly effective in inhibiting LNCaPH tumor growth. On day 70, the average tumor volume for control mice treated with saline was 6.9-fold greater than that measured when treatment was initiated. For mice treated with si-Vav3, the tumor volumes were 5-fold greater and the size of tumors on day 70 were statistically smaller than those of tumors from mice treated with the vehicle control (P < 0.01). Docetaxel significantly inhibited tumor growth, and the tumor volume on day 70 was slightly larger than the average tumor volume determined when treatment was initiated. Tumors from mice treated with si-Vav3 plus docetaxel were statistically smaller than those from mice treated with docetaxel alone (P < 0.01), and the tumor volume on day 70 was 59% smaller than that when treatment was initiated. It appears reasonable to suppose that a lower concentration of docetaxel can be used in combination therapy with si-Vav3 because wide differences were not observed between these two groups despite the statistical significance of the differences. In addition, during a 70-day observation period, we did not note any toxicity in mice treated with si-Vav3 plus docetaxel, as evaluated by their body weights and physical appearance (data not shown). These results in tumor xenografts support the data of the combined effect of si-Vav3 with docetaxel on cancer cell growth *in vitro*.

**Figure 5:** **Effects of Vav3 siRNA (si-Vav3) and docetaxel (DTX) on xenograft tumor growth.** LNCaPH cells implanted subcutaneously into nude mice and treated with si-Vav3 and/or DTX. **A**, dose–response curves of si-Scr and si-Vav3. Changes in the tumor volume were followed over time. The initial tumor volume (n = 8) was considered as 100%, and the average tumor volumes are expressed as percentages of the average initial tumor volume of each group on day 21 after LNCaPH cell inoculation. Values represent the mean ± SE. Asterisk indicates P <0.05 compared with the findings in control tumors. Arrows indicate treatment days. **B***, in vivo* combination study in LNCaPH bearing nude mice. Change in the tumor volume was followed over time. The initial tumor volume (n = 8) was considered as 100%, and the average tumor volumes are expressed as percentages of the average initial tumor volume of each group on day 21 after LNCaPH cell inoculation. Values represent the mean ± SE. Asterisk indicates P <0.05 compared with the findings in control tumors. Arrows indicate treatment days. **C***,* immunoblot analysis of Vav3 in control, si-Scr-treated, and si-Vav3-treated tumors was performed using an anti-Vav3 antibody. Blots were stripped and reprobed with an antibody against β-tubulin. **D**, representative H&E staining (100× magnification) and immunohistochemical analysis of Vav3, Ki-67, pAR, and M30 CytoDeath in xenograft tumor specimens (200× magnification ). **E**, data table lists the mean ± SE for four groups.

The article "Targeting the Vav3 oncogene enhances docetaxel-induced apoptosis through the inhibition of androgen receptor phosphorylation in LNCaP prostate cancer cells under chronic hypoxia" was published in 2013. Journal: Mol Cancer.

On day 70 after inoculation, tumor tissues were harvested from euthanized mice and subjected to immunoblot analysis of Vav3, H&E staining and immunohistochemical staining of Vav3, Ki-67, pAR, and a commercially available cell death marker, M30 CytoDeath. Treatment with si-Vav3 effectively downregulated Vav3 expression compared with its expression level in control and si-Scr-treated tumors, illustrating the effectiveness of intratumoral injection (Figure 5C). Histological evaluation revealed that docetaxel alone or si-Vav3 plus docetaxel caused necrosis in some areas of xenograft tumors (Figure 5D). Significant downregulation of Vav3 staining was observed in tumors from mice treated with si-Vav3 alone or in combination with docetaxel but not in tumors from mice treated with docetaxel alone (Figure 5D). Representative immunohistochemical staining of Ki-67, pAR, and M30 CytoDeath is shown in Figure 5D, and the immunohistochemical findings are summarized in Figure 5E. The mean percentage of Ki-67-positive tumor cells in si-Vav3- or docetaxel-treated tumors was significantly decreased compared with that in control tumors (42 ± 8% and 11 ± 5%, respectively, versus 82 ± 10%, P < 0.005), and an even more significant reduction was observed in tumors treated with si-Vav3 plus docetaxel (7 ± 3%, P < 0.005). A significant decrease in the number of pAR-positive cells was observed in tumors treated with si-Vav3 alone or in combination with docetaxel compared with the number of pAR-positive cells in control tumors (45 ± 9% and 43 ± 9%, respectively, versus 91 ± 3%, P < 0.05) but not in tumors treated with docetaxel alone (89 ± 8%). The average apoptotic index for the control tumors was 0.4 ± 0.1% compared with 8 ± 5% (P < 0.05) and 24 ± 8% (P < 0.005) in tumors from mice treated with si-Vav3 and docetaxel, respectively. Tumors from mice treated with the combination of si-Vav3 and docetaxel exhibited the highest apoptotic index (35 ± 9%), which was significantly greater than that in control tumors (P < 0.005). Compared with the results obtained in tumors from mice treated with docetaxel alone, the Ki-67 labeling (P < 0.05) and apoptotic indices (P < 0.05) and the number of pAR-positive cells (P < 0.05) were all statistically significant in tumors treated with the combination of si-Vav3 and docetaxel.

The article "Targeting the Vav3 oncogene enhances docetaxel-induced apoptosis through the inhibition of androgen receptor phosphorylation in LNCaP prostate cancer cells under chronic hypoxia" was published in 2013. Journal: Mol Cancer.

## Discussion

Docetaxel is a microtubule-targeting drug currently used as a standard first-line chemotherapeutic agent for the management of HRPC that has contributed to improved survival and quality of life in patients with advanced prostate cancer; however, its effectiveness is limited by intolerance and the development of docetaxel-refractory prostate cancer [26-28]. It is therefore reasonable to expect further improvements in treatment outcomes when docetaxel is combined with other therapeutic modalities active against prostate cancer. Because the Vav3 oncogene is overexpressed in androgen-independent prostate cancer, in which it regulates cell growth [16,17], verifying whether Vav3 is a signaling molecule appears beneficial for establishing a new therapeutic target for treating HRPC in combination with docetaxel. We first tested the anti-cancer potential of interrupting the Vav3 signaling pathway using siRNA followed by investigating the impact of si-Vav3 in combination with docetaxel. The goals of this study were to (1) explore Vav3 as a novel therapeutic target for human prostate cancer, (2) define the biological effects of si-Vav3 when combined with docetaxel in human prostate cancer cells in culture and experimental animal models, and (3) characterize the downstream signaling pathways of Vav3 in human prostate cancer cells. This approach allowed us to advance our understanding of the possible importance of Vav3 as an efficacious therapeutic modality for prostate cancer beyond its commonly described associations with cell morphology and transformation.

In the present study, we made certain observations. (1) Vav3 was overexpressed in LNCaP cells cultured under chronic hypoxia (LNCaPH) characterizing androgen independence [25]. (2) Vav3 activated pro-survival signaling pathways, including the activation of PI3K/Akt and ERK, which caused downstream Bad and AR phosphorylation in LNCaPH cells. (3) Downregulation of Vav3 signaling pathways by siRNA in combination with docetaxel significantly inhibited LNCaPH cell growth through the induction of apoptosis *in vitro* and in mouse xenografts *in vivo*. (4) si-Vav3 inhibited the phosphorylation of Akt and ERK, resulting in the inhibition of Bad and AR phosphorylation. (5) Docetaxel also inhibited the phosphorylation of Akt and ERK but activated JNK, resulting in increased Bcl-2 phosphorylation, and decreased Bad phosphorylation. To the best of our knowledge, this is the first report to show that siRNA knockdown of Vav3 can be combined with docetaxel against prostate cancer to yield increased sensitivity *in vitro* and *in vivo*.

The article "Targeting the Vav3 oncogene enhances docetaxel-induced apoptosis through the inhibition of androgen receptor phosphorylation in LNCaP prostate cancer cells under chronic hypoxia" was published in 2013. Journal: Mol Cancer.

Recent studies have suggested controversies in the roles of hypoxic tumor microenvironment in prostate cancer. Dihydrotestosterone increased hypoxia response element (HRE)-mediated transcriptional activity in prostate cancer, and androgen is involved in the response to hypoxia through hypoxia-inducible factor-1α [29]. In addition, castration therapy was reported to decrease the synthesis of vascular growth factors, such as VEGF and angiopoietins, and upregulate hypoxia, leading to apoptosis in prostate cancer [30]. Therefore, androgen deprivation therapy, which induces apoptosis by degenerating the vascular support system of the tumor, is reasonable for androgen-dependent prostate cancer. In contrast, tumor hypoxia is progressively associated with increased AR activity, reduced oxidative defense, genomic instability, and apoptosis resistance, and it may be associated with the transition to androgen independence in prostate cancer [31,32]. Suzuki *et al*. reported that prostate cancer progresses in hypoxic conditions and transforms to the androgen independent state by suppressing the androgen response [33]. Moreover, Butterworth *et al.* also demonstrated that hypoxia could select for androgen-independent prostate cancer cells with more malignant behaviors including invasion and metastasis [34]. In other words, hypoxia may select androgen-independent prostate cancer with a more malignant phenotype. We also previously reported that chronic hypoxia markedly potentiated androgen-independent growth and malignant behavior in LNCaP cells [25]. Hence, it appears important to overcome the hypoxia-induced malignant potential reflecting the androgen-independent state in prostate cancer.

Vav3 has been identified as a Ros receptor protein tyrosine kinase-interacting protein functioning as a signaling molecule downstream of Ros [23]. Vav3 also plays a role in epidermal growth factor receptor-, insulin receptor-, and insulin-like growth factor-mediated signaling pathways [23]. Lyons *et al*. reported that Vav3 expression is elevated in prostate cancer specimens and is coupled to growth factor receptor pathways that are upregulated during the progression of androgen-dependent prostate cancer cells to the androgen-independent state [15]. Because Vav3 expression in LNCaP cells was also increased after long-term androgen deprivation, the possibility that Vav3 expression plays a role in the acquisition of androgen independence was suggested by these observations. Our previous study revealed that androgen-dependent LNCaP cells could acquire androgen independence through Vav3 overexpression when cultured under chronic hypoxia [24,25]. That is, prostate cancer under chronic hypoxia may reflect the androgen independent state with Vav3 overexpression.

The article "Targeting the Vav3 oncogene enhances docetaxel-induced apoptosis through the inhibition of androgen receptor phosphorylation in LNCaP prostate cancer cells under chronic hypoxia" was published in 2013. Journal: Mol Cancer.

We hypothesized that Vav3 may be a key therapeutic target molecule in the regulation of prostate cancer growth and survival under chronic hypoxia. To test this hypothesis, we examined the effects of Vav3 depletion by siRNA on cell growth and downstream cell signaling pathways in LNCaPH cells. We demonstrated that si-Vav3 alone inhibited LNCaPH cell growth and induced apoptosis *in vitro* and in mouse xenografts *in vivo*. These results are consistent with previous observations reported by Dong *et al*., in which Vav3 depletion by siRNA inhibited growth in both androgen-dependent and androgen independent prostate cancer [17]. However, the effect of si-Vav3 was weak and this study was designed to determine the combinatorial effects of docetaxel on cancer cell growth and apoptosis. In this study, we noted that the growth-inhibitory effect of si-Vav3 on LNCaPH cells occurred through a decrease in phosphorylated Akt and ERK, leading to the induction of apoptosis (Figures 2 and 3). Accompanying this apoptotic induction, we observed that si-Vav3 could induce caspase-9 activation (Figure 3) but not casapase-8 activation (data not shown). Taken together, these results suggest that si-Vav3-induced apoptosis mainly depends on mitochondrial pathways rather than death receptor-mediated pathways. In addition, combination treatment significantly decreased the phosphorylation of Akt and ERK and increased the phosphorylation of JNK. This indicates that combined si-Vav3 and docetaxel treatment increased apoptosis by modulating Akt, ERK, and JNK phosphorylation.

si-Vav3 induced the apoptotic activity of the pro-apoptotic member of the Bcl-2 family protein Bad, which is a common target of Akt and ERK [35,36]. We noted that inhibition of survival kinase cascades targeting Bad, including the inhibition of Akt and ERK phosphorylation by si-Vav3, resulted in apoptosis (Figures 2 and 3). In addition, si-Vav3 simultaneously inhibited the androgen signaling mediated by AR, a ligand-activated transcription factor and survival factor. It has been amply documented that AR, PI3K/Akt, and ERK pathways are important features contributing to uncontrolled prostate cancer cell growth and survival. In addition, increased AR activity is caused by crosstalk between AR and multiple intracellular signaling cascades, particularly PI3K/Akt and ERK pathways [17,37]. Consistent with a previous report, Vav3 downregulation inhibited AR phosphorylation through its convergent signaling network of PI3K/Akt and ERK in LNCaPH cells. Because PI3K/Akt and ERK pathways can regulate prostate cancer survival through the AR pathway, we investigated whether inhibiting PI3K/Akt and ERK pathways by kinase-specific inhibitors could affect AR phosphorylation. We found that treatment with LY294002 or U0126 decreased the phosphorylation of AR with a concomitant reduction of Akt and ERK phosphorylation in both LNCaP and LNCaPH cells (Figure 4). Thus, treatment with LY294002 increased apoptosis, whereas the effect of U0126 on cell apoptosis was attenuated compared with that of LY294002 because of the low level of basal ERK activity. Interestingly, the effects of LY294002 on apoptosis was stronger in LNCaPH cells than in LNCaP cells because of the high basal Akt phosphorylation level. Collectively, these results indicate that the PI3K/Akt signaling pathway plays a crucial role in LNCaPH cell growth, although cancer cell growth regulated by Vav3, at least in part, originated from activated ERK signaling. Our observations support the view that the PI3K/Akt pathway, which is activated by Vav3, is mainly involved in AR activity in prostate cancer development and progression [17,38].

The article "Targeting the Vav3 oncogene enhances docetaxel-induced apoptosis through the inhibition of androgen receptor phosphorylation in LNCaP prostate cancer cells under chronic hypoxia" was published in 2013. Journal: Mol Cancer.

In this study, although docetaxel also induced LNCaPH cell apoptosis by the inhibition of Bad phosphorylation including the inhibition of Akt and ERK phosphorylation, the level of AR phosphorylation was unaffected by docetaxel. It has been reported that docetaxel can induce apoptosis by PI3K/Akt inhibition in prostate cancer [39]. Similarly, our findings suggested that Bad phosphorylation is mainly regulated by the PI3K/Akt pathway because basal ERK activity is very low in LNCaPH cells, although ERK phosphorylation is inhibited by docetaxel.

JNK, also called SAPK, is involved in development, morphogenesis, cell differentiation, and cell death in response to various environmental stresses including mitogen growth factors, inflammatory cytokines, oxidative stress, and diverse extracellular stimuli including cytotoxic drugs. Depending on the stimulus and cell type, JNK has essential roles in modulating the function of the mitochondrial pro- and anti-apoptotic proteins, such as Bcl-2 and Bad [40,41]. A previous study demonstrated that the duration and intensity of JNK activation are associated with apoptotic cell death and that Bad dephosphorylation is accompanied by increases in JNK phosphorylation and activity [42]. Moreover, JNK activation leads to inactivation of the survival functions of Bcl-2 through Bcl-2 phosphorylation [43]. In this study, Bad dephosphorylation and Bcl-2 phosphorylation with an elevation of JNK phosphorylation were induced by docetaxel, suggesting that JNK positively regulates apoptosis induction through Bad dephosphorylation and Bcl-2 phosphorylation.

## Conclusions

In summary, this study demonstrated that Vav3-mediated signaling converges with PI3K/Akt, ERK, and AR signaling pathways in support of the growth and survival of prostate cancer cells under chronic hypoxia. Because the pAR-positive cell ratio was not found to be associated with apoptosis and tumor growth delay in *in vivo* analysis, LNCaPH cell growth appeared to be regulated by both AR-dependent and AR-independent pathways. Therefore, si-Vav3, which targets the PI3K/Akt, ERK, and AR signaling axis, was effective when combined with docetaxel, which targets Bcl-2 and Bad. Increased Bad and AR phosphorylation by the activation of PI3K/Akt and ERK signaling pathways upon Vav3 stimulation contributes to prostate cancer growth under chronic hypoxia (Figure 6A), whereas increased Bcl-2 phosphorylation and decreased Bad phosphorylation through the activation of JNK signaling by docetaxel coupled with decreased phosphorylation of Bad and AR through the inhibition of PI3K/Akt and ERK signaling pathways upon the addition of si-Vav3 contributes to increased apoptosis (Figure 6B). The present study describes a potentially useful approach of utilizing the combination of docetaxel and si-Vav3 to enhance the apoptosis of prostate cancer cells under chronic hypoxia. In addition, docetaxel plus si-Vav3 exhibited no toxicity in mice, which makes it an attractive and safe therapeutic strategy in future clinical application to treat prostate cancer. This approach may provide a novel strategy for the treatment of HRPC, particularly advanced prostate cancer in which the Vav3 signaling pathway is activated.

**Figure 6:** **Proposed molecular mechanisms of Vav3-mediated signaling pathways in LNCaPH cells. A**, following the induction of Vav3 expression under chronic hypoxia, Vav3 can phosphorylate Bad at Ser 112 and AR at Ser 81 through PI3K/Akt and ERK pathways, resulting in cancer cell survival. **B**, Vav3 siRNA can inhibit Vav3-mediated signaling pathways and docetaxel can phosphorylate Bcl-2 at Ser 70 and dephosphorylate Bad through JNK and PI3K/Akt pathways, respectively, and thus, these two signaling pathways can merge to activate the caspase cascade, resulting in apoptosis.

The article "Targeting the Vav3 oncogene enhances docetaxel-induced apoptosis through the inhibition of androgen receptor phosphorylation in LNCaP prostate cancer cells under chronic hypoxia" was published in 2013. Journal: Mol Cancer.

## Methods

### Cell culture and hypoxia induction

LNCaP human prostate cancer cells were maintained in RPMI 1640 medium supplemented with 10% heat-inactivated fetal bovine serum (FBS) (Bio-Whittaker, Walkersville, MD, USA), 50 IU/ml penicillin, and 50 μg/ml streptomycin (GibcoBRL, Grand Island, NY, USA) and cultured at 37°C in a humidified atmosphere of 5% CO_2_. To establish chronic hypoxia-conditioned LNCaP (LNCaPH) cells, LNCaP cells were cultured under hypoxia (1% O_2_) for 6 months. The experiments using LNCaPH cells were performed under hypoxic conditions. KPK13 human renal cell carcinoma cells were cultured in minimum essential medium (MEM) (GibcoBRL) supplemented with 10% FBS, with 50 IU/ml penicillin, and 50 μg/ml streptomycin in 5% CO_2_ at 37°C.

### Immunocytochemistry

Cultured cells were washed with PBS, fixed in methanol for 20 min, and incubated in 10% goat normal serum (Nichirei, Tokyo, Japan) for 10 min at 37°C. Cells were incubated in a primary antibody against Vav3 (1:50 dilution; Epitomics, Burlingame, CA, USA) at room temperature in PBS with 1% BSA for 60 min. After incubation with the primary antibody, the secondary antibody fluorescein dye (Alexa Fluor 488)-conjugated goat anti-rabbit IgG (1:40 dilution) (Invitrogen, Carlsbad, CA, USA) was added in PBS with 1% BSA for 30 min. Cells were visualized using confocal laser microscopy followed by nuclear staining with 1 μg/ml 2,4-diamidino-2-phenylindole dihydrochloride n-hydrate (Dojindo, Kumamoto, Japan).

### Transient transfection of Vav3 siRNA

Cells were transiently transfected with a Vav3 siRNA duplex (si-Vav3; final concentration of 60 nmol/l) or a control siRNA (a random scrambled sequence: si-Scr; final concentration of 60 nmol/l) using Lipofectamine RNAiMAX (Invitrogen) according to the manufacturer’s instructions. The sequence of the siRNA against Vav3 synthesized by Invitrogen is 5^′^- AUAUUCUCCUGACUCUUUGGUCCUG(dT)(dT)-3^′^. Following transfection, cells were subjected to growth inhibition, live/death, flow cytometric, and immunoblot analyses.

### Growth inhibition assay

Cell viability was determined using a cell proliferation assay. In brief, exponentially growing cells were seeded in 6-well plates at 1 × 10^5^ cells/well. After overnight culture, the culture medium was changed to fresh standard medium containing 5 nM docetaxel (Sigma, St. Louis, MO, USA) for 0–72 h or various concentrations of docetaxel (0, 1, 2.5, and 5 nM) for 72 h in the presence or absence of si-Vav3. After treatment, the cell number was counted with a hemocytometer.

The article "Targeting the Vav3 oncogene enhances docetaxel-induced apoptosis through the inhibition of androgen receptor phosphorylation in LNCaP prostate cancer cells under chronic hypoxia" was published in 2013. Journal: Mol Cancer.

### Live/death analysis

Cells were treated with si-Vav3, 5 nM docetaxel, or si-Vav3 plus 5 nM docetaxel for 48 h. Live and dead cells were detected using the Live/Death Viability/Cytotoxicity assay kit (Molecular Probes, Eugene, OR) for which fluorescence was observed and pictures were taken at 4× magnification. The data from three independent experiments were expressed as a mean percentage.

### Flow cytometric and DNA fragmentation analyses

For cell cycle analysis, flow cytometric analysis of propidium iodide-stained nuclei was performed. In brief, cells treated with si-Vav3, 5 nM docetaxel, or si-Vav3 plus 5 nM docetaxel for 0–72 h or various concentrations of docetaxel (0, 1, 2.5, and 5 nM) for 72 h in the presence or absence of si-Vav3 were plated at a density of 5 × 10^5^ cells in a 60-mm dish overnight. The cells were collected by trypsinization and fixed with 70% ethanol. The fixed cells were incubated with 100 μg/ml RNase A (Sigma) for 30 min and stained with 25 μg/ml propidium iodide (Chemicon, Temecula, CA, USA) for 30 min. Cell cycle distribution was analyzed with a FACScan flow cytometer and CellQuest software (Becton Dickinson Labware, Lincoln Park, NJ, USA). The data from three independent experiments were expressed as a mean percentage. The apoptotic response was also measured by the Cell Death Detection ELISA^PLUS^ photometric enzyme immunoassay for the quantitative determination of cytoplasmic histone-associated DNA fragments (Roche, Indianapolis, IN, USA). In brief, the cytoplasmic fractions of the untreated control cells and cells treated with si-Scr, si-Vav3, 5 nM docetaxel, or si-Vav3 in combination with 5 nM docetaxel were transferred to a streptavidin-coated plate and incubated for 2 h at room temperature with a mixture of peroxidase-conjugated anti-DNA and biotin-labeled antihistone. The plate was washed thoroughly and incubated with 2, 2^′^-azino-di[3-ethylbenzthiazolin-sulfonate]. The absorbance was measured at 405 nm with a reference wavelength of 492 nm.

### Cytotoxicity assay

To determine the involvement of PI3K/Akt, ERK, and c-jun N-terminal kinase (JNK) pathways in cell apoptosis, cells were treated with LY294002 (Calbiochem, Darmstadt, Germany), U0126 (Calbiochem), or SP600125 (Sigma), respectively, for 48 h. Control cells were cultured in the presence of an equivalent amount of DMSO as a vehicle.

The article "Targeting the Vav3 oncogene enhances docetaxel-induced apoptosis through the inhibition of androgen receptor phosphorylation in LNCaP prostate cancer cells under chronic hypoxia" was published in 2013. Journal: Mol Cancer.

### Immunoblot analysis

Protein was extracted from cell pellets with a lysis buffer (50 mM Tris, pH 8.0, 150 mM NaCl, 0.02% NaN_3_, 0.1% SDS, 1% NP-40, 0.5% sodium deoxycholate, and 1 mM PMSF) in the presence of a protease inhibitor cocktail (Roche Applied Science, Indianapolis, IN, USA). Samples containing equal amounts of protein (30 μg) were electrophoresed on 8–16% Tris-glycine gels (Invitrogen) and transferred to nitrocellulose membranes. After blocking with T-TBS containing 5% nonfat milk powder, the membranes were incubated with mouse monoclonal antibody against phospho-Akt (Ser 473) (1:1000 dilution; Cell Signaling, Danvers, MA, USA), phospho-ERK (Thr 202/Tyr 204) (1:1000 dilution; Cell Signaling), phospho-stress−activated protein kinase (SAPK)/JNK (Thr 183/Tyr 185) (1:1000 dilution; Cell Signaling), and Bcl-2 (1:1000 dilution; Santa Cruz Biotechnology, Santa Cruz, CA, USA), or rabbit polyclonal antibodies against Vav3 (1:1000 dilution; Cell Signaling), Akt (1:1000 dilution; Cell Signaling), ERK (1:1000 dilution; Santa Cruz Biotechnology), phospho-Bcl-2 (Ser 70) (1:1000 dilution; Cell Signaling), Bad (1:1000 dilution; Cell Signaling), phospho-Bad (Ser 136) (1:1000 dilution; Cell Signaling), ERK (1:1000 dilution; Cell Signaling), SAPK/JNK (1:1000 dilution; Cell Signaling), AR (1:1000 dilution; Millipore, Temecula, CA), phospho-AR (Ser 81) (1:500 dilution; Millipore), caspase-3 (1:1000 dilution; Cell Signaling), caspase-9 (1:500 dilution; Cell Signaling), or poly(ADP-ribose) polymerase (PARP) (1:1000 dilution; Cell Signaling) at 4°C overnight. After washing with T-TBS, the membranes were incubated with corresponding secondary antibodies, which were conjugated with horseradish peroxidase (Santa Cruz Biotechnology). The blots were stripped and reprobed with anti-β-tubulin antibody (1:5000 dilution; Sigma). Immunoreactive bands were visualized with ECL plus (Amersham Pharmacia Biotech, Little Chalfont, UK) and quantified by scanning densitometry using NIH Image software (version 1.55).

### Formation of siRNA/atelocollagen complex

Atelocollagen is a type I collagen of calf dermis that is highly purified by pepsin treatment (Koken Co., Ltd, Tokyo, Japan). The siRNA and atelocollagen complexes were prepared as follows. An equal volume of atelocollagen (in PBS at pH 7.4) and siRNA solution was combined and mixed by rotation at 4°C for 20 min. The final concentration of atelocollagen *in vivo* was 0.5%.

### In vivo animal experiment

Four-week-old male athymic nude mice (20–24 g; BALB/*c nu/nu* mice) were housed in accordance with and approved by the Institutional Animal Care and Use Committee of Oita University. For subcutaneous injection, LNCaPH cells were trypsinized, and single-cell suspensions (2 × 10^6^ cells) were mixed 1:1 with Matrigel and then injected into both flanks. To determine the optimal concentration of the siRNA/atelocollagen complex, dose–response tests including si-Scr as a vehicle control and si-Vav3 were performed. Three weeks after the injection of mice with LNCaPH cells, when the tumor volume reached 100 mm^3^, the mice were randomly divided into seven treatment groups (non-treatment; 0.5 μg, 2.5 μg, and 10 μg of si-Scr/tumor; 0.5 μg, 2.5 μg, and 10 μg of si-Vav3/tumor), each consisting of four mice. The siRNA/atelocollagen complex was injected directly into the tumors once a week for 7 consecutive weeks. Tumor size was quantified by measuring in two dimensions with calipers, and tumor volume was calculated every 7 days according to the equation (*l* × *w*^2^)/2, where *l* = length and *w* = width. The mice were monitored daily for changes in weight and other signs of acute toxicity. After optimizing the concentration of the siRNA/atelocollagen complex (2.5 μg siRNA/50 μl/tumor), the effects of combination therapy with docetaxel was assessed. Tumor cell-bearing mice were randomly divided into four treatment groups (si-Scr, si-Vav3, docetaxel, and docetaxel + si-Vav3), each consisting of four mice. An intratumoral injection of the siRNA/atelocollagen complex (si-Vav3 or si-Scr) was performed with or without docetaxel 10 mg/kg i.p. once weekly for 7 consecutive weeks. When treatments were completed, animals were sacrificed, and tumor tissues were harvested for immunoblot analysis, H&E staining and immunohistochemistry.

The article "Targeting the Vav3 oncogene enhances docetaxel-induced apoptosis through the inhibition of androgen receptor phosphorylation in LNCaP prostate cancer cells under chronic hypoxia" was published in 2013. Journal: Mol Cancer.

### Immunohistochemical protocol

After sacrifice, s.c. tumor tissues were fixed with 10% buffered formalin and embedded in paraffin. The formalin-fixed, paraffin-embedded tissues were cut to 4-μm sections and deparaffinized in xylene followed by treatment with a graded series of ethanol and rehydration in PBS. The sections were incubated in 0.3% H_2_O_2_ for 10 min to inactivate endogenous peroxidase, followed by washing in PBS. To block non-specific binding to sections and eliminate non-specific staining, 10% normal goat serum in PBS was applied and incubated for 10 min. The following primary antibodies were used: Vav3, Ki-67 (DAKO, Carpinteria, CA, USA), phospho-AR (pAR) (Abnova, Thaipei, Taiwan), and M30 CytoDeath (Roche Applied Science, Mannheim, Germany). They were diluted 50×, 1×, 100×, and 50×, respectively, with PBS containing 1% BSA. After washing with PBS, sections were incubated with secondary antibodies, which were conjugated with peroxidase-labeled amino acid polymer (DAKO). The immune complex was visualized using a 3,3′-diaminobenzidine peroxytrichloride substrate solution (DAKO). Slides were then counterstained with hematoxylin and mounted. The evaluation of Ki-67, pAR, and M30 CytoDeath staining was based on the proportion of positive-stained cells among a total of 1000 cells that were counted in five randomly selected areas.

The article "Targeting the Vav3 oncogene enhances docetaxel-induced apoptosis through the inhibition of androgen receptor phosphorylation in LNCaP prostate cancer cells under chronic hypoxia" was published in 2013. Journal: Mol Cancer.

### Statistical analysis

Values were expressed as means ± SE. Statistical analysis was performed using Student’s *t*-test. The limit for statistical significance was set at P <0.05.

## Abbreviations

AR: Androgen receptor; siRNA: Small interfering RNA; PI3K: Phosphatidylinositol 3-kinase; JNK: c-jun N-terminal kinase; Bcl-2: B-cell lymphoma 2; Bad: Bcl-xL/Bcl-2-associated death promoter; HRPC: Hormone-refractory prostate cancer; GTPase: Rho guanosine triphosphatase; GEF: Guanine nucleotide exchange factor; ERK: Extracellular signal-regulate kinase; FBS: Fetal bovine serum; MEM: Minimum essential medium; PARP: poly(ADP-ribose) polymerase; HRE: Hypoxia response element.

## Competing interests

The authors declare that they have no competing interests.

## Authors’ contributions

TN, MY, FS and HM designed this study and performed all experiments with the help of KH, TI and RS. KM, MM and HM critically read the manuscript and gave good advice. TN wrote this manuscript. All authors read and approved final manuscript.
